# Analysis of the Effect of Sichs on Gastric Ulcer Rats Based on RNA Sequencing Technique

This article has been retracted.

**DOI:** 10.1155/2022/9325836

**Published:** 2022-06-13

**Authors:** Lin Su, Hong Song, Ti Ren, Wen Chen, Jiaqi Zhang, Guiyue Wang, Junfang Yang, Xin Hou, Yan Shen, Xiaogu Liu

**Affiliations:** ^1^Department of Traditional Chinese Medicine Diagnosis, Zhejiang Chinese Medical University, Hangzhou, Zhejiang 310053, China; ^2^Department of Rehabilitation Ward III, Hospital of Zhejiang People's Armed Police, Hangzhou, Zhejiang 310053, China

## Abstract

**Objective:**

To research the mechanism of action and transcriptomic characteristics for the intervention effect of self-made Chaihuang decoction (Sichs) on gastric ulcer (GU) rats with liver qi stagnation and spleen deficiency and to clarify the therapeutic pathway and effective target.

**Methods:**

Thirty SD rats were randomly divided into the control group, model group, and Sichs group (10 rats per group). The model of GU rats with liver qi stagnation and spleen deficiency was established through multifactor compound simulation of traditional Chinese medical (TCM) etiology and acetic acid method. Histopathological changes in the gastric antrum tissue were observed with H&E staining. RNA sequencing (RNA-seq) was utilized to check differentially expressed genes (DEGs) in the gastric antrum tissues of rats, and gene ontology (GO) and KEGG pathway enrichment analyses were performed. The key DEGs were validated using qRT-PCR.

**Results:**

Sichs could ameliorate gastric antrum tissue injury in GU rats with liver qi stagnation and spleen deficiency. After RNA-seq, it was found that Sichs could reverse 225 upregulated genes and 26 downregulated genes in the model group. And the DEGs between the Sichs group and the model group were related to cell division, complement activation, and phospholipase A2 (Pla2g2a) activity. According to KEGG pathway analysis, DEGs between the two groups were mainly enriched in signaling pathways such as cell cycle, p53 signaling pathway, and linolenic acid metabolism. The validation results of the four key DEGs were consistent with the analysis trend of sequencing results.

**Conclusion:**

Sichs can effectively improve GU with liver qi stagnation and spleen deficiency in rats through the signaling pathways related to cell cycle and lipid metabolism.

## 1. Introduction

Gastric ulcer (GU), resulting in damage or necrosis of gastric mucosa, is a digestive system disease induced by a variety of factors (such as stress, helicobacter pylori infection, and taking nonsteroidal anti-inflammatory drugs) [1, 2]. And GU belongs to the gastric abscess and stuffiness of the stomach in traditional Chinese medical science (TCM). The incidence of GU is 20-60 cases per 100,000 people with 5%-10% of mortality worldwide [3]. Some studies have indicated that patients with long-term GU have a higher risk of the occurrence of gastric cancer. The occurrence of GU is caused by multiple factors, such as the interference of acids, pepsin, cholic acid, helicobacter pylori, ethanol, and nonsteroidal anti-inflammatory drugs to defense factors [4]. In TCM, emotional disorders and stagnation of liver qi are considered to be main causes of GU. Due to the side effects and drug resistance of traditional drugs (clarithromycin, amoxicillin, omeprazole, etc.) in the treatment of GU, it is still necessary to find new therapeutic methods [5].

Self-made Chaihuang decoction (Sichs) is a Chinese medicine formula with the effects of replenishing Qi and invigorating spleen, soothing liver, and activating blood circulation and can effectively treat GU in clinical practice [6]. Studies have also found that Sichs could effectively promote GU-injured gastric mucosa healing [7–9]. However, there are no intensive studies on the mechanism of action of GU.

Transcriptome analysis based on RNA sequencing (RNA-seq), a technology which utilizes high-throughput sequencing methods to observe cells, has become increasingly mature with the development of science and technology [10]. RNA-seq has become an indispensable tool for transcriptome-wide analysis of differentially expressed genes (DEGs) and differential splicing. Currently, RNA-seq is widely applied to elucidate different physiological and pathological conditions and to study the molecular mechanisms of drug action [11]. Some studies have analyzed the molecular mechanism of the effect of Lindera reflexa Hemsl on relieving GU in rats using RNA-seq [12]. In view of the large number of components, the complexity of therapeutic effects, and unclear mechanism of action of the TCM, this study adopted RNA-seq to identify the DEGs of Sichs. And according to transcriptomics, the mechanism of action of Sichs was further explored.

## 2. Materials and Methods

### 2.1. Experimental Drugs

In Radix et Rhizoma Rhei preparation solution, Radix et Rhizoma Rhei was broken into powder and then was soaked with distilled water. Subsequently, a 4-hour water bath was performed at 50°C. After removing the drugs, the medicinal juice was kept. Then, 1 ml/100 g gavage was conducted.

In Sichs, 12 g Radix Bupleuri, 12 g Radix Astragali, 18 g Radices Paeoniae Alba, 12 g Giant knotweed root, 9 g Cassia Twig, and 12 g Rhizoma Cyperi were prepared [6] (all drugs were conformed to the standard of *Pharmacopoeia of the People's Republic of China* (2020)). The concentrated decoction of the drug is 1 g/1 ml. After removing the dregs, the juice was collected and stored at 4°C in the fridge. The dosage of the drugs in rats was calculated based on the equivalent dose between adults and rats, which was 6.25 times of the adult dose (containing 0.76 g/kg of crude drugs) [13].

### 2.2. Experimental Animals

A total of 30 SPF-grade SD rats (weight: 150-180 g) were purchased from Shanghai Lab. Animal Research Center (Production license No.: SCXK (Hu) 2013-0016). The rats were housed in a barrier environment with 23 ± 1°C of ambient temperature and 50%-65% of relative humidity in the Animal Experimental Center of Zhejiang Chinese Medical University. Complete nutrient pellet feed and water were provided for the rats ad libitum.

### 2.3. The Establishment of the Model of Gastric Ulcer Rats with Liver Qi Stagnation and Spleen Deficiency

The model of GU rats with liver qi stagnation and spleen deficiency was established with multifactor compound simulation of TCM etiology and acetic acid method [14, 15]. Radix et Rhizoma Rhei preparation solution was administered at 1 ml/100 g daily in the morning, and the middle of the rat tail was clamped with a wooden clip for 30 min/rat. Every afternoon, a fuse with a weight of 10% of the body weight of the rat was wrapped at the base of the rat's tail. And then, the rats were placed in a tank with a water depth of 50 cm and a water temperature of 28°C for swimming, to the degree of exhaustion, that is, the tip of the rat's nose was submerged for 10 s. The above trial lasted for 14 days. After fasting for 24 hours on the 15^th^ day, laparotomy was performed under pentobarbital sodium anesthesia (Merck KGaA, Germany). Specifically, the abdominal cavity of the rat was open to expose the corpora ventriculi; then, 0.005 ml/site of 50% glacial acetic acid was injected into the glandular site. After that, corpora ventriculi was returned and the abdominal cavity was closed. Then, the fasting continued, but the water was allowed. Thirty SD rats were randomly divided into the following groups (10 rats per group). In the control group, the rats were gavaged with normal saline. In the model group, after the mole was established successfully, the rats were gavaged with normal saline. In the Sichs group, after the mole was established successfully, the rats were administered 10 mg/kg of Sichs for 14 consecutive days. On completion of the last administration, the fasting was continued but the water was allowed for 24 h. Then, the rats were sacrificed and the blood from the heart and gastric antrum tissues in each group were collected for the subsequent trial.

### 2.4. Evaluation Method for Reconstructed Rat Model

The model evaluation methods mainly include general condition observation, pathological observation, and verification of serum level of liver qi stagnation and spleen deficiency [16]. (1) With *Zhong Yi Shi Yan Dong Wu Mo Xing Fang Fa Xue* (a book that summarized experimental animal model methodology of Traditional Chinese Medicine) as a reference, the criteria of the general condition observation were shown as follows: Rats had the symptoms of fatigue and lassitude, food intake reduction, slow weight gain, dull hair, irritability, and soft and loose stools. (2) The criteria for pathological observation were displayed as follows: Significant ulcerative changes occurred in gastric histopathological sections. (3) The criteria for the liver qi stagnation was shown as follows: The level of noradrenalin (NE) in the serum of the control group was lower while the level of serum 5-hydroxytryptamine (5-HT) was higher compared with the model group. The criteria for the spleen deficiency were displayed as follows: The serum gastrin (GAS) level in the control group was higher than that in the model group.

### 2.5. Hematoxylin and Eosin (H&E) Staining

Tissues of the gastric antrum were fixed in 4% paraformaldehyde buffer for 48 h, dehydrated, 3 *μ*m thick sections, and stained with H&E. Subsequently, histopathological changes were observed under the microscope.

### 2.6. Biochemical Assays

The serum levels of NE, 5-HT, and GAS were measured by ELISA kits (Nanjing Jiancheng Bioengineering Institute, Jiangsu, China). Briefly, all serum samples were processed according to the instructions of each ELISA kit. OD values were measured at 450 nm using an enzyme marker.

### 2.7. RNA-Seq

Total RNA was first isolated and purified with TRIzol (Invitrogen, America), and then, the amount and purity of total RNA were measured with NanoDrop ND-1000. The integrity of the RNA was tested by Bioanalyzer 2100, and the verification was conducted through agarose electrophoresis. Validation criteria were shown as follows: concentration > 50 ng/*μ*l, RIN > 7.0, OD260/280 > 1.8, and total RNA > 1 *μ*g. After reverse transcription of total RNA into cDNA, E. coli DNA polymerase I (New England Biolabs, America) was applied for double-strand synthesis. Specifically, the complex duplex of DNA and RNA was converted into a DNA duplex, and at the same time, dUTP solution was incorporated into the duplex to supplement the ends of the duplex. And the A nucleobases were added at the ends of the double-stranded DNA to link with T nucleobases. Then, the fragment sizes were screened and purified with magnetic beads. After the duplex was digested by Uracil-DNA Glycocasylase (UDG) (New England Biolabs, America), libraries with a fragment size of 300 bp ± 50 bp were formed through PCR. Finally, with PE150 as the sequencing mode, double-end sequencing was performed according to the instructions of the Illumina NovaSeq™ 6000 kit.

### 2.8. Identification of DEGs

A gene was defined as a DEG using the “limma” package of R software [17] between two groups, when the adjusted *P* value was < 0.05 and the gene expression fold change (FC) value was ≥1 or <-1, which were visualized as volcano plots.

### 2.9. Gene Ontology (GO) and Kyoto Encyclopedia of Genes and Genomes (KEGG) Pathway Enrichment Analyses

We used DAVID (https://david.ncifcrf.gov/) [18] to carry out GO functional annotation and KEGG pathway enrichment analyses on the DEGs. An adjusted *P* value < 0.05 was considered statistically significant [19].

### 2.10. qRT-PCR

Approximately 50–100 mg of tissue samples were taken out to grind fully, and then, total RNA was extracted with the TRIzol single-step RNA isolation method. Further, after 20 *μ*l of DEPC was added for resuspension, the concentration and purity test was conducted. Then, total RNA was reverse transcribed into cDNA using a reverse transcription kit (Takara, Japan). The quantitative fluorescence PCR solution was prepared according to the instructions of PCR kit (Takara, Japan), and the PCR was performed with a quantitative fluorescence PCR instrument. The reaction conditions were shown as follows: 95°C for 30 s, 95°C for 5 s, and 60°C for 30 s, a total of 41 cycles. Three replicated wells were set for each sample, the experiment was repeated three times, and the CT value of each well was recorded. The relative expression of genes was calculated using 2^−*ΔΔ*Ct^. The primers used in this experiment were designed and synthesized by Shanghai Sangon Biotech. The primer sequences were displayed in Table 1.

### 2.11. Statistical Analysis

Statistical analysis of experimental data was performed using SPSS 24.0 software (IBM, Chicago, USA), and the results were expressed as mean ± standard deviation (SD). *T*-test analysis was utilized for comparison between two groups, and one-way analysis of variance (one-way ANOVA) for comparison among multiple groups. *P* < 0.05 was considered to be a significant difference criterion.

## 3. Results

### 3.1. Sichs Can Improve Gastric Tissue Injury in Gastric Ulcer Rats with Liver Qi Stagnation and Spleen Deficiency

Firstly, the model of GU rats with liver qi stagnation and spleen deficiency was evaluated. According to the results of the detection of serum index in rats, the NE content in the model group was significantly increased compared with the control group, while the GAS and 5-HT contents were significantly decreased (Figure 1(a)). The above results indicated that the model was established successfully. In experimental session, rats in the control group had bright coat color, flexible posture, moderate fecal quality, and increasing body weight with flat trend. Rats in the model group had dark coat color, irritable temper, and slow weight gain after modeling. Compared with the control group at the same stage, the rats in the model group showed emaciation and a very significant difference in body weight change after completion of modeling. After modeling for 10 days, the swimming time of rats in the model group was significantly shortened, and even could not swim with weight bearing, and appeared in huddled together, arched back, debilitating, and irritability. And some rats had positive tail-pulling defecation response, dirty anus, and pale mucosa in the nasal tip and foot web. After Sichs intervention treatment for 14 days, the above conditions were significantly improved than before. Treated rats have a flexible posture, increased food intake, increased body weight, dry fecal texture, and gradually regain luster in coat color (Figure 1(b).

Further examination of the histopathological structure of the antrum revealed that, in the control group, the mucosal layer and intrinsic glands remained intact, and the morphology of chief cells, parietal cells, and myxocytes was regular, without edema fluid, inflammatory cell infiltration, or fibrous hyperplasia. In the model group, a large number of inflammatory cells were infiltrated, the defect reached the mucosa, the intrinsic glands were disorganized, and the morphology of chief cells, parietal cells, and mucinous cells was irregular. Compared with the model group, the glands were arranged neatly, the cell morphology was more regular, and only a small range of benign proliferative changes was observed on the surface of the gastric mucosa in the Sichs group (Figure 1(c)). The above results indicated that Sichs could notably improve gastric tissue injury in GU rats with liver qi stagnation and spleen deficiency.

According to the naked eye observation, gastric mucosa in the control group was smooth. The color was soft and glossy, and there were many coating solutions. The mucosal wrinkles were regular and complete, and the gastric wall elasticity was good. The surface color of gastric mucosa in the model group was pale, the surface mucus was less, and mucosal edema or erosion was observed. Most of the ulcer surfaces or bleeding points of different sizes were found, and the elasticity of gastric wall was poor. After 14 days of medication or saline, the improvement of the model group was not obvious, and the Sichs group recovered better (Figure 1(d)).

### 3.2. DEG Screening

RNA-seq technology was further adopted to study the mechanism of Sichs in the treatment of GU with liver qi stagnation and spleen deficiency. According to the results of the analysis, there were 2355 DEGs (*P* < 0.05) between the model group and the control group, including 2147 upregulated genes and 208 downregulated genes. There were 823 DEGs (*P* < 0.05) between the Sichs group and the model group, including 370 upregulated genes and 453 downregulated genes (Figure 2(a)). Further, the differential genes in the volcano diagram were plotted again with the Wayne diagram. The result revealed that the Sichs group reversed 251 DEGs in the model group, including 225 upregulated genes and 26 downregulated genes (Figure 2(b)).

### 3.3. Functional Analysis of DEGs among Three Groups

GO and KEGG enrichment analyses were performed to analyze 251 differential genes reversed by Sichs. The results of the analysis indicated that a total of 58 GO entries were enriched for DEGs, including 29 biological processes, 21 cellular components, and 8 molecular functions. Enriched GO biological process entries involved cell division, complement activation, negative regulation of endopeptidase activity, and lipoxygenase pathway. GO cellular component entries included the cytoplasm, extracellular region, spindle pole, and kinesin complex. GO molecular function entries involved phospholipase A2 activity, endopeptidase inhibitor activity, and structural molecule activity (Figures 3(a) and 3(b)). Besides, pathway enrichment of differential genes mainly involved the cell cycle, p53 signaling pathway, glycerophospholipid metabolism, alpha-linolenic acid metabolism, arachidonic acid metabolism, linoleic acid metabolism, ether lipid metabolism, staphylococcus aureus infection, and complement and coagulation cascades (Figure 3(c)).

### 3.4. Validation of Four Key DEGs' Level

It was found based on the results of KEGG pathway enrichment analysis of reversed genes that Pla2g2a and Pla2g4f genes were involved in multiple lipometabolism-related pathways, such as arachidonic acid metabolism, alpha-linolenic acid metabolism, linoleic acid metabolism, and glycerophospholipid metabolism. Ccnb1 and Cdk1 genes were involved in cell cycle signaling pathways and P53 signaling pathways were associated with cell cycle, cell growth, and apoptosis. Therefore, in this experiment, the above four genes were selected for the validation of sequencing analysis results. The results of validation suggested that, compared with the model group, the mRNA expression level of Pla2g4f, Pla2g2a, Cdk1, and Ccnb1 in the Sichs group was notably downregulated (Figure 4). The change trend of validation results was consistent with the sequencing results.

## 4. Discussion

GU is a common disease in clinical practice, with an incidence of about 10% of the population [20]. However, the incidence of GU has increased due to lifestyle changes in recent years, and a risk of further deterioration may occur in patients without prompt treatment. Fan et al. [21] concluded that the reason why GU can result in precancerous gastric lesions is that the mucosa at the ulcer margin is more prone to intestinal metaplasia in order to adapt to changes in the internal environment and resist the stimulation of harmful factors. Moreover, patients with GU and gastritis are often accompanied by Helicobacter pylori infection, and Helicobacter pylori infection is one of the important factors in the occurrence of precancerous gastric lesions. Yang et al. [22] found that the proapoptotic factor level was higher in tissues of GU with precancerous gastric lesions than that in tissues without precancerous lesions. Some other studies have pointed out that GU is a risk factor for precancerous gastric lesions, and the proapoptotic factor level in patients with precancerous gastric lesions is higher than that in patients without precancerous lesions [23].

According to the recordation of *Zheng Meng-Qian Cheng* (a famous ancient Chinese book written by Zhang Zai), the normal physiological activities of the human body are inseparable from the balances formed by adjusting qi movement, the interaction and oppositional constraint of Yin and Yang. GU belongs to gastric abscess and stuffiness of stomach in the theories of TCM. And after summarizing the previous experience and long-term clinical observation, we found that liver qi stagnation and spleen deficiency are the main pathogenesis and pathological attributes of GU [15, 24]. The Sichs used in this experiment was modified by adding Radix Bupleuri, Rhizoma Cyperi, and Rhizoma Polygoni Cuspidati on the basis of Huangqi Jianzhong decoction, with a significant clinical application effect. Huangqi Jianzhong decoction is a famous prescription for tonifying deficiency. Specifically, in the prescription, Radix Astragali and Cassia Twig, sweet and warming drugs, can dredge liver qi; the addition of Rhizoma Polygoni Cuspidati can relieve pain and remove blood stasis. In brief, the whole prescription can dredge liver qi, invigorate spleen, regulate qi, promote blood circulation, and remove blood stasis. The results of this study also showed that Sichs significantly improved gastric tissue injury in GU rats with liver qi stagnation and spleen deficiency.

RNA-seq technology, which studies the regulation of gene transcription at the molecular level, can identify the main action pathways of drugs by comparing the gene expression among the three groups. In this experiment, the RNA-seq technique was utilized to sequence the transcriptome of gastric antrum tissues from rats in the control group, model group, and Sichs group, respectively. And then, the process of gene content change in gastric antrum ulcer of the rat model of GU with liver qi stagnation and spleen deficiency under the intervention of Sichs was determined. Through deep mining and analysis of DEGs in the model group reversed by Sichs, it was found that DEGs were mainly enriched in pathways related to cell cycle regulation and lipid metabolism.

Cell cycle regulation, a bidirectional regulatory mechanism, is critical for balancing cell proliferation and apoptosis. Pardee [25] believed that each link in the process of cell cycle regulation contributed to the dynamic balance of maintaining the unity of opposites between Yin and Yang. Several studies have shown that gastric disease progression and the development of neoplastic diseases can be effectively intervened through cell cycle regulation. Xu et al. [26] and other studies found that the intervention of Chaishao Liujun decoction on chronic atrophic gastritis (CAG) rats with liver qi stagnation and spleen deficiency is mainly achieved by inhibiting the excessive proliferation of gastric mucosal cells and balancing the level of cell proliferation and apoptosis. And the mechanism of action of Chaishao Liujun decoction is associated with the inhibition of high expression of c-Myc, P53, PCNA, and Ag-NOR. Li et al. [27] found that Jiawei Qifang Weitong granules can downregulate CDK2\4 gene expression to inhibit tumor cell division and proliferation, thereby reversing the progression of precancerous lesions of gastric cancer. In this study, Sichs affected the cell cycle regulation mainly through the cell cycle pathway and P53 signaling pathway. And the DEGs of Ccnb1 (cyclin B1) and Cdk1 (cyclin-dependent kinase) showed different degrees of high expression in the model group. Ccnb1 is a cell cycle-related gene, and Cdk1 is a key regulatory enzyme in cell cycle progression. The combination of Ccnb1 and Cdk1 can activate CDKs and produce specific complexes, thereby prompting cells to enter the S phase from the G1 phase, accelerating the rate of cell proliferation, and shortening the cell cycle [28]. The experimental results showed that the expression level of Ccnb1 and Cdk1 decreased to a different extent after the intervention of Sichs. The result above indicated that Sichs could inhibit cell proliferation and achieve effective regulation of cell cycle by downregulating the expression of Ccnb1 and Cdk1 genes, thereby balancing Yin and Yang in the organism.

The lipid metabolic pathways affected by Sichs mainly include glycerophospholipid metabolism, alpha-linolenic acid metabolism, arachidonic acid metabolism, and linoleic acid metabolism. Pla2g2a and Pla2g4f, the differential genes of the experiment, had high expression in above lipid metabolic pathways. Pla2g2a and Pla2g4f, from the phospholipase A2 family (PLA2), are low molecular weight extracellular enzymes. More specifically, Pla2g2a and Pla2g4f are involved in the regulation of phospholipid metabolism in biofilms by the hydrolysis of calcium ion-catalyzed sn-2 ester bond of phosphoglyceride and the release of free fatty acids and lysophosphatide. Xing et al. [29] found a positive correlation between the Pla2g2a expression and drug resistance of human gastric cancer progression. Additionally, Pla2g2a is a direct target of Wnt/*β*-catenin signaling in human gastric cancer [30]. And Sichs can significantly reduce the high expression of Pla2g2a and Pla2g4f genes.

In summary, through the signaling pathways related to cell cycle regulation and lipid metabolism, Sichs can regulate cell division and proliferation as well as fatty acid metabolism and ester metabolism to restore the balance of Yin and Yang of the organism, thereby treating GU with liver qi stagnation and spleen deficiency.

## Figures and Tables

**Figure 1:** Effects of Sichs on gastric tissue injury in GU rats with liver qi stagnation and spleen deficiency. (a) ELISA was utilized to check the levels of noradrenalin (NE), gastrin (GAS), and 5-hydroxytryptamine (5-HT) in the serum of rats in each group. (b) Body weight changes in rats in each group. (c) H&E staining was applied for the detection of histopathological structure of gastric antrum in rats of each group. (d) The gastric mucosa of the rats in each group: ^∗∗^*P* < 0.01 vs. the control group, ^##^*P* < 0.01 vs. the model group.

**Figure 2:** RNA-seq analysis of differential genes among the three groups. (a) Volcano diagram of differential genes among three groups: the ordinate represented the statistical significance of the difference in gene expression change; the abscissa represented the fold changes in differential expression of genes in different samples; the blue represented downregulated significant DEGs; the red represented upregulated significant DEGs, and dots in gray represented nonsignificant DEGs. (b) Differential gene Wayne diagram among three groups.

**Figure 3:** GO and KEGG pathway enrichment of DEGs. (a, b) GO enrichment barplot (a) and GO enrichment scatterplot (b) for biological function analysis of DEGs. (c) KEGG pathway enrichment scatterplot for DEGs.

**Figure 4:** Sichs significantly declines the expression levels of the key DEGs. The mRNA expressions of Pla2g2a, Pla2g4f, Ccnb1, and Cdk1 in the gastric antrum tissues were detected by qRT-PCR. ^∗∗^*P* < 0.01 vs. the model group.

**Table 1:** Primer sequences.

Gene name	Sequence (5′-3′)
Pla2g2a	F: 5′-CATTGTGGTGTGGGTGGCAGAG-3′
	R: 5′-CGGTAGGAGAACTTGTAGGTCAGAAAC-3′
Pla2g4f	F: 5′-TCCCAGCGACCTTTATCTTTCACATG-3′
	R: 5′-CTTGCTTCCTCCATCTTGCTAGTCTG-3′
Ccnb1	F: 5′-AAGTCAGCGAACAGTCAAGAATACCC-3′
	R: 5′-AGGTTCAGGCTCAGGCTCATCC-3′
Cdk1	F: 5′-CAGTTCATGGATTCTTCGCTCGTTAAG-3′
	R: 5′-ATCTGCCAGTTTGATTGTTCCTTTGTC-3′

## Data Availability

The data used to support the findings of this study are available from the corresponding author upon request.
